# LncRNA SNHG7 promotes pancreatic cancer proliferation through ID4 by sponging miR-342-3p

This article has been retracted.

**DOI:** 10.1186/s13578-019-0290-2

**Published:** 2019-03-22

**Authors:** Dongfeng Cheng, Juanjuan Fan, Yang Ma, Yiran Zhou, Kai Qin, Minmin Shi, Jingrui Yang

**Affiliations:** 1 Pancreatic Disease Center, Department of General Surgery, Rui Jin Hospital Affiliated to Shanghai Jiao Tong University School of Medicine, No.197 Rui Jin Er Road, Shanghai, China; 2 Yichuan Community Health, Shanghai, China; 3 Research Institute of Digestive Surgery, Ruijin Hospital, Shanghai Jiaotong University School of Medicine, Shanghai, China

**Keywords:** LncRNA SNHG7, Pancreatic cancer, MiR-342-3p, ID4

## Abstract

**Background:**

Small nucleolar RNA host gene 7 (SNHG7) is a novel identified oncogenic gene in tumorigenesis. However, the role that SNHG7 plays in pancreatic cancer (PC) remains unclear. In this study, we aimed to investigate the functional effects of SNHG7 on PC and the possible mechanism.

**Methods:**

The expression levels of SNHG7 in tissues and cell lines were measured by RT-qPCR. Cell viability, apoptosis, migration and invasion were examined to explore the function of SNHG7 on PC. Bioinformatics methods were used to predict the target genes. The mechanism was further investigated by transfection with specific si-RNA, miRNA mimics or miRNA inhibitor. Tumor xenograft was carried out to verify the effects of SNHG7 in vivo.

**Results:**

We found that SNHG7 was overexpressed in both PC tissues and cell lines. High expression level of SNHG7 was correlated with the poor prognosis. SNHG7 knockdown inhibited the proliferation, migration and invasion of PC cells. Moreover, SNHG7 was found to regulate the expression of ID4 via sponging miR-342-3p. Additionally, this finding was supported by in vivo experiments.

**Conclusions:**

LncRNA SNHG7 was overexpressed in PC tissues, and knockdown of SNHG7 suppressed PC cell proliferation, migration and invasion via miR-342-3p/ID4 axis. The results indicated that SNHG7 as a potential target for clinical treatment of PC.

## Background

Pancreatic cancer (PC) is one of the deadliest human malignancies in digestive tract, exhibiting a 5-year survival rate of less than 5% [1]. The most common options for PC treatment are surgical resection and systemic chemo-radiotherapy. However, because of the early metastasis, the prognosis is poor. Therefore, there is an urgent need to understand the molecular mechanisms underlying PC progression [2].

LncRNAs, a kind of non-coding RNAs with more than 200 nt in length, are reported to play roles in a variety of human cancers, including PC [3–6]. For example, HOTTIP, MALAT1 and MEG3 are regarded as important regulators of tumor progression [7]. Small nucleolar RNA host gene 7 (SNHG7), a lncRNA located on chromosome 9q34.3 with a length of 2157 bp, is a novel identified oncogenic gene functioning in different types of human cancers, including breast cancer, bladder cancer, colorectal cancer and prostate cancer [8–11]. However, little is known about the role of SNHG7 in PC.

MicroRNAs, a class of non-coding RNAs with a length of ~ 22 nt, regulate the expression of target genes by binding the 3′-UTR of mRNAs [12]. MiRNAs are reported to function in the progression of different cancers [13–15]. An increasing study has demonstrated that lncRNAs are likely to function as competing endogenous RNAs (ceRNAs) via sponging miRNAs, thereby regulating the specific target gene of miRNA. For example, it was found that SNHG7 was upregulated in prostate cancer tissues, and played as a ceRNA to regulate the cycle progression and acted as an oncogenic gene through sponging miR-503 [11]. However, the interaction between SNHG7 and miRNAs in pancreatic cancer has not been reported.

In this study, we found that SNHG7 was over-expressed in PC tissues and cell lines, and associated with poor prognosis in PC patients. We also demonstrated that SNHG7 knockdown inhibited PC cell proliferation and metastasis in vitro, as well as suppressed tumor growth in vivo. Moreover, SNHG7 acted as a ceRNA of miR-342-3p and thereby regulate the target gene expression of inhibitor of DNA binding 4 (ID4). Taken together, SNHG7 may serve as a potential target for PC treatment.

## Materials and methods

### Clinical samples

PC tissues and adjacent normal ones were obtained from forty patients undergone cancer resection between 2016 and 2018 at Rui Jin Hospital Affiliated to Shanghai Jiao Tong University School of Medicine. The clinicopathologic characteristics were presented in Table 1.  Informed consents were obtained from every patient before surgery and the procedure of this research had been approved by the Ethics Committee of Rui Jin Hospital Affiliated to Shanghai Jiao Tong University School of Medicine (IRB number: RJEC-2018-087).

**Table 1:** Relationship of LncRNA SNHG7 expression and clinical variables among 40 pancreatic cancer patients

Characteristics	Number (total n = 40)	SNHG7 expression		P value
		High (n = 27)	Low (n = 13)	
Age (years)				
≥ 60	24	16	8	0.802
< 60	16	11	5	
Gender				
Male	25	17	8	0.683
Female	15	10	5	
TNM stage				
I–II	21	11	10	0.021*
II–IV	19	16	3	
Lymph-node metastasis				
Negative	17	9	8	0.028*
Positive	23	18	5	
Tumor size (cm)				
> 2	26	20	6	0.032*
≤ 2	14	7	7	
Tumor differentiation				
Well	6	3	3	0.016*
Moderate	17	10	7	
Poor	17	14	3	

* P < 0.05, the difference is significant

### Cell culture

PC cell lines (AsPC-1, BxPC-3, SW1990, PANC-1 and PaCa-2), normal pancreatic duct epithelial cell line (HPDE6-C7) and HEK293T cell line were purchased from American Type Culture Collection (ATCC, USA). All cell lines were cultured in Dulbecco’s modified Eagle’s medium (DMEM, Invitrogen) supplemented with 10% FBS at 37 °C in 5% CO_2_.

### Cell transfection

LncRNA SNHG7 siRNA (si-SNHG7) and negative control (si-NC) were purchased from GenePharma (Shanghai, China). Mir-342-3p mimics, miR-342-3p inhibitor and corresponding negative controls were purchased from Sangon Biotech (Shanghai, China). Lipofectamine 2000 (Thermo Fisher Scientific, Waltham, USA) was used for transfection.

### RNA isolation and quantitative PCR

Total RNA was isolated from tissues as well as cells using Trizol reagent (Invitrogen), according to the manufacturer’s protocol. cDNA was synthesized from RNA (100 ng) of each sample by a PrimeScript RT reagent kit (RR047A, TaKaRa, Japan). Real-time quantitative PCR was performed with SYBR PremixEx Taq kit (RR420A, TaKaRa) according to the manufacturer’s protocol. U6 and β-Actin were used as internal controls. Relative expression was calculated by the 2^−ΔΔCq^ method and every experiment was performed in triplicate. The sequences of Real-time PCR primers were listed in Table 2.

**Table 2:** Primers of qRT-PCR

Gene	Primers
SNHG7	
Forward	5′-CGATACCATTGAACACGCTGC-3′
Reverse	5′-GGTTGAGGGTCCCAGTG-3′
miR-342-3p	
Stem-loop primer	5′-GCGCGTGAGCAGGCTGGAGAAATTAACCACGCGCACGGGT-3′
Forward	5′-TCTCACACAGAAATCGC-3′
Reverse	5′-GAGCAGGCTGGAGAA-3′
ID4	
Forward	5′-CGATGAAGGCGGTGAGCC-3′
Reverse	5′-CCAGGCTGTGGATCTTCGT-3′
β-Actin	
Forward	5′-CTCCATCCTGGCCTCGCTGT-3′
Reverse	5′-GCTGTCACCTTCACCGTTCC-3′

### Cell counting kit-8 (CCK-8) assay

CCK-8 assay was performed to detect the cell viability. In brief, transfected cells were maintained in 96-well plates and CCK-8 solution was added into each well. The cell viability was tested every 24 h according to the manufacturer’s instructions at 450 nm.

### Wound healing assay

Wound healing assay was performed to examine the cell migration. In brief, when transfected cells maintained in 6-well plates reached 90–95% confluence, a micropipette tip was used to create a scratch. After 24 h, an X71 inverted microscope (Olympus, Tokyo, Japan) was used to observe the recovery state of the wounds.

### Transwell invasion assays

Transfected cells were seeded in the upper chamber of medium coated with Matrigel. The lower chamber was filled with medium plus with 10% FBS. Twenty-two hours after transfection, 70% ethanol was added into the lower surface of the filter for 20 min, and then 0.1% crystal violet was used to stain the invaded cells for 10 min. The invaded cells were observed in 5 randomly selected fields using a X71 inverted microscope (Olympus, Japan). The whole experiment was completed within 24 h of transfection.

### Luciferase reporter assay

SNHG7 with miR-342-3p binding sites (wild type) or mutant sequences (mutant) were inserted into the pRL-TK plasmid vector (Promega), forming SNHG7-WT and SNHG7-MUT luciferase reporter plasmids. Cells maintained in 96-well plates were co-transfected with luciferase reporter plasmids and miR-342-3p mimics or negative controls. After 48-h incubation, the relative luciferase activities were detected.

### Western blot

After transfection for 48 h, cells were subjected to RIPA lysis buffer (Beyotime) and total protein was exacted. Quantified via a BCA Assay Kit (Pierce, Appleton, WI), equal amounts of each sample were loaded and separated by 10% SDS-PAGE, followed by transferring to PVDF membranes. The PVDF membranes were blocked with 5% non-fat milk for 2 h, and then incubated in specific primary antibodies including ID4 (1:1000, Abcam) and β-Actin (1:3000, Abcam) at 4 °C overnight. Then the membranes were incubated in corresponding HRP-conjugated secondary antibodies for 1 h, after 3 washes with TBST buffer. Lastly, Positive signals were developed by an ECL Kit (GE Healthcare, Freiburg, DE).

### Animal experiments

Female BALB/C nude mice (4 week old) were obtained from Shanghai Experimental Animal Center of Chinese Academy of Sciences (Shanghai, China). PANC-1 cells were stably transfected with sh-SNHG7 and negative control (sh-NC) and injected into the posterior flank of mice. Each group includes 6 mice. The volume of tumor was recorded every week for 5 weeks. After the last measurement, mice were euthanized and the tumor tissues were used for the following analysis of miR-342-3p and ID4 expression levels.

### Immunohistochemical staining

ID4 was detected by incubation in a mouse monoclonal antibody (1:400, Abcam) overnight at 4 °C. After washed with PBS, the sections were incubated in anti-mouse IgG labeled with biotin (1:200) (Beyotime, Jiangsu, China) at 37 °C for 1 h and then with avidin-labeled HRP (Beyotime). The EnVision system (Dako, Glostrup, Denmark) was used to visualize the immunostaining. Four sections were counted in each group membrane or cytoplasm was stained.

### Statistical analysis

All data were expressed as mean ± standard deviation (SD) from at least three repeated experiments. SPSS 17.0 (IBM, Armonk, NY, USA) were used for statistical tests. Student’s *t* test was used to determine the difference between two groups. One-way analysis was used for multiple comparison correlation analysis was determined using Pearson correlation coefficient (r). P < 0.05 was considered to be statistically significant.

## Results

### SNHG7 was upregulated in PC tissues and cell lines

Forty-paired PC and adjacent normal tissues were used to detect the expression levels of SNHG7 by qPCR. Results demonstrated that the SNHG7 expression level was increased in PC tissues, compared with that in normal ones (Fig. 1a). Moreover, the expression levels of SNHG7 were also increased in PC cell lines, compared with that in normal pancreatic cells (HPDE6-C7) (Fig. 1b). Further, Kaplan–Meier analysis revealed that the PC patients with higher SNHG7 expression had poor prognosis than that with low SNHG7 expression (Fig. 1c).

**Fig. 1:** LncRNA SNHG7 was upregulated in pancreatic cancer (PC) tissues and cell lines. **a** Relative expression levels of lncRNA SNHG7 in PC tissues and adjacent normal ones were measured by RT-qPCR. **b** Relative expression levels of lncRNA SNHG7 in human PC cell lines (BxPC-3, AsPC-1, AW1990, PANC-1 and PaCa-2) and normal pancreatic cell line (HPDE6-C7) were determined by RT-qPCR. **c** Kaplan-Meier analysis of overall survival time in PC patients with high and low SNHG7 expression levels. **P < 0.01, compared with normal tissue group or HODE6-C7 group

### SNHG7 knockdown suppressed PC cell proliferation, migration and invasion in vitro

To detect whether SNHG7 played roles in PC, we transfected SNHG7 siRNA or negative control into PANC-1 and PaCa-2 cell lines. As shown in Fig. 2a, SNHG7 expression was significantly decreased after 48 h of transfection, confirming the knockdown efficiency of SNHG7 siRNA. Moreover, SNHG7 knockdown inhibited cell viability, while induced cell apoptosis. To further investigate the function of SNHG7 in PC metastasis, wound healing and transwell assays were performed to determine the cell migration and invasion. Results showed that the migration rate and invasion numbers of PC cells were markedly decreased after si-SNHG7 transfection (Fig. 2d, e).

**Fig. 2:** SNHG7 knockdown suppressed PC cell proliferation, migration and invasion in vitro. After transfection with siRNA of SNHG7 or negative control (NC) into PANC-1 and PaCa-2 cell lines, **a** the expression level of SNHG7 was measured by RT-qPCR; **b** cell viability was determined by CCK-8 assay; **c** the apoptotic rate was measured by flow cytometric; **d** cell migration rate was analyzed by wound healing assay; **e** cell invasion was determined by transwell assay. *P < 0.1, **P < 0.01, compared with si-NC group

### miR-342-3p was a direct target of SNHG7

Accumulating evidence has suggested that lncRNAs are likely to function as competing endogenous RNAs (ceRNAs) by sponging miRNAs. Herein, we predicted miR-342-3p as a potential target of SNHG7 via StarBase software. Figure 3a showed the predicted complementary binding sites, and the luciferase reporter assay confirmed the prediction (Fig. 3b). RT-qPCR revealed that SNHG7 knockdown significantly increased the miR-342-3p expression levels in both cell lines (Fig. 3c). However, SNHG7 showed no obvious change after miR-342-3p mimics transfection (Fig. 3d). Further, the expression levels of miR-342-3p were detected in vivo. As Fig. 3e shown, the miR-342-3p expression level was markedly lower in PC tissue than that in normal ones. Pearson’s correlation analysis revealed that SNHG7 was negatively correlated to miR-342-3p expression in PC tissues (Fig. 3f).

**Fig. 3:** SNHG7 targeted miR-342-3p directly. **a** Schematic representation of binding sites between SNHG7 and miR-342-3p predicted by StarBase software. **b** Luciferase reporter assay was performed after co-transfection with reporter plasmid and miRNAs into HEK293T cells. **c** After transfection with siRNA of SNHG7 or negative control (NC), the expression level of miR-342-3p was measured by RT-qPCR. **d** After transfection with miR-342-3p mimics or miRNA negative control (miR-NC), SNHG7 expression level was measured by RT-qPCR. **e** The expression levels of miR-342-3p in PC tissues and adjacent normal ones were determined by RT-qPCR. **f** Negative correlation between SNHG7 and miR-342-3p in PC tissues. **P < 0.01, compared with miR-NC group, si-NC group or normal tissue group

### SNHG7 knockdown inhibited PC cell proliferation, migration and invasion via miR-342-3p in vitro

Our previous results demonstrated that SNHG7 played roles in PC cell proliferation and metastasis, and SNHG7 interacted with miR-342-3p. Thus, we wanted to investigate whether miR-342-3p was involved in the SNHG7 function on PC cell biological behaviors. The expression level of miR-342-3p was markedly downregulated after miR-342-3p inhibitor transfection, confirming the knockdown efficiency of miR-342-3p inhibitor. Next, miR-342-3p inhibitor or negative control was co-transfected with si-SNHG7, and the cell proliferation, cell migration and cell invasion were assessed. As shown in Fig. 4b, c, miR-342-3p inhibitor mitigated the changes induced by si-SNHG7 in cell viability and cell apoptosis. Additionally, the alterations in cell migration and cell invasion induced by si-SNHG7 were also alleviated by miR-342-3p inhibitor (Fig. 4d, e). The quantitative analysis was presented in Fig. 4f.

**Fig. 4:** SNHG7 promoted PC cell proliferation, migration and invasion via miR-342-3p in vitro. **a** After transfection with miR-342-3p inhibitor or negative control (NC), the expression levels of miR-342-3p in PANC-1 and PaCa-2 cell lines were measured by RT-qPCR. After transfection with si-SNHG7 in the presence of miR-342-3p inhibitor or negative control (NC), **b** cell viability was measured by CCK-8, **c** the apoptotic rate was determined by flow cytometry, **d** cell migration was determined wound healing assay and **e** cell invasion was determined by transwell assay. **f** Quantitative analysis of cell viability, apoptotic rate, migration rate and invasion cell number. **P < 0.01, compared with si-NC group or si-NC + miR-NC group. ^##^< 0.01, compared with si-SNHG7 + miR-NC group

### ID4 was a direct target of miR-342-3p

With the help of TargetScan software, we predicted ID4 as a potential target of miR-342-3p. The putative binding sites were shown in Fig. 5a, which was confirmed by luciferase reporter assay (Fig. 5b). Western blot also demonstrated that the ID4 protein level was downregulated after miR-342-3p mimics transfection (Fig. 5c, d). Moreover, the expression levels of ID4 in vivo were detected. Results showed that the ID4 expression level was significantly overexpressed in PC tissues, compared with that in adjacent normal ones (Fig. 5e). Pearson’s correlation analysis revealed that miR-342-3p was negatively correlated to ID4 expression in PC tissues (Fig. 5f).

**Fig. 5:** ID4 was a direct target of miR-342-3p in PC. **a** Schematic representation of binding sites between miR-342-3p and ID4 predicted by TargetScan software. **b** Luciferase activity assay was performed after co-transfection with reporter plasmid and miRNAs into HEK293T cells. **c**, **d** The protein levels of ID4 in PANC-1 and PaCa-2 cell lines were determined by western blot with transfection of miR-342-3p or negative control. **e** The expression mRNA levels of ID4 in PC tissue sand adjacent normal ones were determined by RT-qPCR. **f** Negative correlation between miR-342-3p and ID4 in PC tissues. **P < 0.01, compared with miR-NC group

### SNHG7 positively regulated the expression of ID4 via miR-342-3p

Subsequently, we wanted to explore whether SNHG7 regulated ID4. Results showed that SNHG7 knockdown induced a marked decrease of ID4 in PC cells, while downregulation of miR-342-3p mitigated the changes in mRNA and protein levels (Fig. 6a–c). In addition, the expression levels of SNHG7 and ID4 in PC tissues showed negative correlation (Fig. 6d).

**Fig. 6:** SNHG7 upregulated ID4 by sponging miR-342-3p in PC. After transfection with si-SNHG7 in the presence of miR-342-3p inhibitor or negative control (miR-NC), **a** the ID4 mRNA expression level was measured by RT-qPCR; **b**, **c** the ID4 protein expression level was measured by western blot. **d** Positive correlation between SNHG7 and ID4 in PC tissues. **P < 0.01, compared with si-NC + miR-NC group; ^##^P < 0.01, compared with si-SNHG7 + miR-NC group

### SNHG7 knockdown suppressed PC tumorigenesis in vivo

We further investigated the function of SNHG7 on PC tumorigenesis in vivo. PANC-1 cells transfected with sh-SNHG7 or negative control were injected into the posterior fank of the mice. The tumor volume of each mouse was measured weekly. As demonstrated in Fig. 7a, b, SNHG7 knockdown decreased the tumor volume and weight compared with negative control. Moreover, the expressions of miR-342-3p was upregulated and ID4 was downregulated in tumor tissues from sh-SNHG7 group, compared with that in sh-NC group (Fig. 7b–e).

**Fig. 7:** SNHG7 knockdown suppressed PC tumorigenesis in vivo. PANC-1 cells transfected with sh-SNHG7 or negative control (sh-NC) were injected into the posterior fank of mice, 7 day later, **a** the tumor volume of each mouse was measured weekly; **b** miR-342-3p expression level was measured by RT-qPCR; **c**, **d** ID4 protein level was determined by western blot. **e** ID4 expression level was detected by immunohistochemical staining. **P < 0.01, compared with sh-SNHG7 group

## Discussion

Increasing study has indicated the important roles of lncRNAs in tumorigenesis or metabolic disorders [16]. SNHG7 has been reported as an oncogene functioning in several kinds of cancers. For example, Li et al. found that SNHG7 promoted colorectal cancer progression by acting as a ceRNA of miR-34a and thereby increasing GALN7 expression level [10]. SNHG7 could also accelerate prostate cancer proliferation via miR-503/Cyclin D1 pathway [11]. In this study, we demonstrated that SNHG7 was overexpressed in PC tissues as well as cell lines. Consistently, high expression of SNHG7 in PC patients was related to shorter survival. Moreover, SNHG7 knockdown suppressed PC cell proliferation, migration and invasion, indicating the oncogenic role of SNHG7 in PC tumorigenesis.

Accumulating lncRNAs were reported to perform as ceRNAs by competing for shared microRNAs. For instance, recently, Dong et al. demonstrated that lncRNA TINCR accelerated epithelial-mesenchymal transition via sponging miR-125b in breast cancer [17]. Zhang et al. showed that PCA3 regulated prostate cancer by targeting miR-218-5p and HMGB1 [18]. As to SNHG7, Ren et al. revealed that SNHG7 promoted glioblastoma progression by suppressing miR-5095 [19]. Luo et al. reported that SNHG7 regulated breast cancer via miR-186 [8]. To investigate the mechanism of SNHG7 regulating PC, we focused on the cross-regulation between miRNAs and SNHG7. Since miR-342-3p has been reported as tumor suppressors in a series of cancers. For instance, miR-342-3p downregulation promoted hepatocellular carcinoma growth both in in vitro and in vivo [20]. Xue et al. showed that overexpression of miR-342-3p suppressed the proliferation and migration of non-small cell lung cancer cells [21]. Thus, we focused on miR-342 which is one of the potential targets of SNHG7 predicted by software and investigated whether miR-342-3p mediated the effects of SNHG7 on PC progression. Results showed that miR-342-3p was the target of SNHG7, and miR-342-3p suppression could mitigate the inhibitory effects on PC cell proliferation and metastasis induced by si-SNHG7.

MiRNAs are known to downregulate gene expressions by base-pairing with the 3′-UTR of targeted mRNAs [22]. For example, mirR210 promoted lung adenocarcinoma proliferation and metastasis by targeting LOXL4 [23]. MiR-342 regulated breast cancer progression via modulating ID4 [24]. Holger et al. found that miR-335 suppressed breast cancer by targeting ID4 [25]. The ID genes, first identified in 1990, were reported to play important roles in normal development and in cancer [26]. ID4, a member of the ID family, has attracted increasing attention due to its heterogeneous roles in different cancer types [27]. Studies on the function of ID4 in various tumor types displayed controversial. Kuzontkoski et al. demonstrated that ID4 was upregulated in glioblastoma multiforme and promoted angiogenesis and growth [28]. Beger et al. demonstrated that ID4 played roles in BRCA1 regulatory pathway and thus might promote the tumorigenic potential of cells in breast cancer and ovarian cancer [29]. On the contrary, ID4 was considered as a putative tumor suppressor with decreased expression levels in several types of cancers. For example, ID4 was found down-regulated in prostate cancer due to promoter hypermethylation [30]. Agnes et al. showed that the downregulation of ID4 by promotor hypermethylation might contribute to gastric adenocarcinoma [31].

In this study, we discovered that ID4 was overexpressed in PC tissues, and SNHG7 positively regulated ID4 via miR-342 in PC cells. Up to now, the most prevalent interaction mode for lncRNAs is that they act as sponges to downregulate the target miRNAs expression levels, and thus mitigate the suppression of miRNAs on their target genes. For instance, Zhang et al. showed that ID4 promoted cell proliferation in hepatocellular carcinoma [32]. Notably, Crippa et al. demonstrated that miR-342 regulated BRCA1 expression by modulating ID4 in breast cancer [24]. In the current study, we found that ID4 was overexpressed in PC tissues and cell lines, and had a negative correlation with miR-342-3p. Moreover, SNHG7 positively regulate the expression of ID4 in vitro, which could be mitigated by miR-342-3p.

## Conclusions

Taken together, we identified SNHG7 as an oncogene that play important roles in PC cell proliferation, migration and invasion. In terms of mechanism, SNHG7 could positively regulate ID4 by sponging miR-342-3p. The findings of this study indicated that SNHG7/miR-342-3p/ID4 axis might be an efficient therapeutic approach for PC.
